RETRACTED

# The cellular source for APOBEC3G's incorporation into HIV-1

**DOI:** 10.1186/1742-4690-8-2

**Published:** 2011-01-06

**Authors:** Jing Ma, Xiaoyu Li, Jian Xu, Quan Zhang, Zhenlong Liu, Pingping Jia, Jinming Zhou, Fei Guo, Xuefu You, Liyan Yu, Lixun Zhao, Jiandong Jiang, Shan Cen

**Affiliations:** 1 Institute of Medicinal Biotechnology, Chinese Academy of Medical Science, Beijing, PR China; 2 State Key Laboratory for Molecular Virology and Genetic Engineering, Institute of Pathogen Biology, Chinese Academy of Medical Science, Beijing, PR China; 3 Lady Davis Institute for Medical Research and McGill AIDS Centre, Jewish General Hospital, Montreal, Quebec, Canada; 4 Microbiology & Immunology, McGill University, Montreal, Quebec, Canada

## Abstract

**Background:**

Human APOBEC3G (hA3G) has been identified as a cellular inhibitor of HIV-1 infectivity. Viral incorporation of hA3G is an essential step for its antiviral activity. Although the mechanism underlying hA3G virion encapsidation has been investigated extensively, the cellular source of viral hA3G remains unclear.

**Results:**

Previous studies have shown that hA3G forms low-molecular-mass (LMM) and high-molecular-mass (HMM) complexes. Our work herein provides evidence that the majority of newly-synthesized hA3G interacts with membrane lipid raft domains to form Lipid raft-associated hA3G (RA hA3G), which serve as the precursor of the mature HMM hA3G complex, while a minority of newly-synthesized hA3G remains in the cytoplasm as a soluble LMM form. The distribution of hA3G among the soluble LMM form, the RA LMM form and the mature forms of HMM is regulated by a mechanism involving the N-terminal part of the linker region and the C-terminus of hA3G. Mutagenesis studies reveal a direct correlation between the ability of hA3G to form the RA LMM complex and its viral incorporation.

**Conclusions:**

Together these data suggest that the Lipid raft-associated LMM A3G complex functions as the cellular source of viral hA3G.

## Background

Human APOBEC3G (hA3G) has been identified as one of anti-HIV-1 host factors [1]. hA3G belongs to an APOBEC superfamily containing at least 11 members, which share a cytidine deaminase motif (a conserved His-X-Glu and Cys-X-X-Cys zinc coordination motif) [2]. The APOBEC superfamily in humans includes APOBEC1, APOBEC2, APOBEC3A-H (hA3A-H), APOBEC4 and activation-induced cytidine deaminase (AID). The virus counters hA3G's anti-viral activity through the viral protein Vif (virion infectivity factor), which interacts with cytoplasmic hA3G as a part of Vif-Cul5-SCF complex, resulting in the ubiquitination and degradation of hA3G [3,4].

Viral encapsidation of hA3G is an essential step for its antiviral activity. Only if hA3G is encapsidated into the virions, can it exert its antiviral activity on the replication of progeny virons in the infectious target cells. This encapsidation of hA3G is facilitated by HIV-1 Gag. The nucleocapsid (NC) domain of Gag mediates the interaction of Gag with hA3G [5-9]. Although the Gag/hA3G interaction has been investigated extensively [10-12], the cellular source of viral hA3G remains unclear. It was found that hA3G in the HIV-1 virion was not reduced as much as the cellular hA3G in the presence of Vif. Furthermore, our previous work has also shown that the removal of the C-terminal region of hA3G results in a significant decrease in its cellular concentration without a corresponding decrease in its incorporation into viral particles [6]. These observations suggest that viruses may recruit hA3G from a particular intracellular pool, and the decrease in total cellular hA3G does not reflect any change occurring in this pool which acts as cellular source of viral hA3G.

RETRACTED

The main cytoplasmic form of hA3G in H9 and 293T cells has been reported to be an enzymatically inactive, high-molecular-mass (HMM) ribonucleoprotein complex [13]. RNase treatment converts this complex to an enzymatically active, low-molecular-mass (LMM) form [13]. Biochemical studies have demonstrated the HMM hA3G complex associates with several cellular RNA binding proteins, as well as certain mRNAs and small non-coding RNAs [14-16]. hA3G has been shown to dynamically associate with various RNPs including ribosomes, miRNA-induced silencing complexes, RoRNPs, processing bodies, stress granules, and Staufen granules [14,16].

Recent work suggests that HIV-1 recruits hA3G from the cellular pool of newly-synthesized enzymes prior to its assembly into the HMM RNA-protein complexes, because of the appearance of viral hA3G shortly after its synthesis [17]. In favor of this hypothesis, most components of the HMM hA3G complex have not been found in virions containing hA3G. In addition, Khan *et al*. reported that encapsidation of hA3G into HIV-1 virions involves lipid raft association and does not correlate with hA3G oligomerization [18]. Nevertheless, another group showed that hA3G mutants failing to form the HMM complex were poorly incorporated into the HIV-1 particle, suggesting that the HMM hA3G may act as the cellular source for virion encapsidation [19].

The purposes of this study are to better characterize cellular distribution of hA3G, and provide insight into the cellular source for hA3G encapsidation into HIV-1. Our work herein shows that the majority of newly-synthesized hA3G interacts with lipid rafts, and acts as both the precursor of mature HMM hA3G complex and the cellular source of hA3G in HIV-1.

RETRACTED

## Results

### The subcellular distribution of hA3G in P100 and S100 fractions

We first analyzed the cytoplasmic distribution of hA3G, using a subcellular fractionation assay. H9 cells, a human T-cell line expressing endogenous hA3G, were lysed by dounce homogenization in hypotonic TE buffer in the presence of RNase inhibitor and protease inhibitor. Similarly, 293T cells that do not express endogenous hA3G were transfected with a plasmid coding for HA (hemagglutinin) tagged hA3G, and then lysed 48 hours post-transfection. Following centrifugation of the cell homogenate at low speed to remove nuclei and unbroken cells, the resultant supernatant (S1) was ultra-centrifuged at 100,000 × g, resulting in pellet (P100) and supernatant (S100). Western blots of the P100 and S100 fractions were probed with either anti-hA3G or anti-HA for the samples derived from H9 cells or 293T cells, respectively (Figure 1A). Approximate 85% of total endogenous hA3G in H9 cells presented in the P100 (lanes 1 to 3), and a similar pattern was also obtained from hA3G transiently expressing in 293T cells (lane 4 to 6). Next, we analyzed the S1, P100 and S100 fractions prepared from 293T cells expressing hA3G, using a 4-35% discontinuous Opti-prep velocity gradient. Nine fractions were collected from the top to the bottom of the gradient, and then subjected to Western blot. In these gradients, hA3G in the S1 was found in both LMM fractions (including fractions 3 and 4) and HMM fractions (including fractions 7 and 8), as shown in the top panel of Figure 1B. hA3G in the P100 was solely detected in fractions 7 and 8 (middle panel, Figure 1B), and co-sediments with the HMM form of hA3G found in the S1, while hA3G in the S100 was only found in fractions 3 and 4 (bottom panel, Figure 1B). These results suggest that the majority of hA3G in the P100 and S100 fractions represented the HMM and LMM forms of hA3G respectively.

**Figure 1:** **The cellular distribution of hA3G in P100 and S100 fractions**. H9 cells and 293T cells expressing HA tagged hA3G were lysed in hypotonic TE buffer, and the resultant S1 was ultra-centrifuged, resulting in the P100 and the S100 fractions. The S1, P100 and S100 fractions prepared from 293T cells were analyzed by using a 4-35% discontinuous Opti-prep velocity gradient, as described in Methods. **A**. Western blots of the S1, P100, and S100 fractions were probed with either anti-hA3G (left) or anti-HA (right) for the samples derived from H9 cells or 293T cells, respectively. **B**. Nine fractions were collected from the top to the bottom of the gradient, then subjected to Western blot probed with anti-HA. The fraction numbers increase from the top to the bottom of the gradient.

RETRACTED

### Steady state hA3G in the cytoplasm appears in three different forms

hA3G has been shown to localize to lipid rafts, which are specialized membrane domains enriched in certain lipids, cholesterol and a specific set of proteins [5]. We reasoned that some of the HMM form of hA3G might result from association of soluble hA3G with lipid rafts. To examine this, P100 was further analyzed by floatation assay. After ultra-centrifugation at 100,000 × g overnight in sucrose gradient, all the collected fractions were subjected to Western Blot probed with anti-Caveolin-1 (lipid raft marker), anti-membrane transferrin receptor (TFR, a cytoplasm membrane bound protein) and anti-HA. As shown in Figure 2A, total HMM hA3G was fractionated into raft (lane 3 and 4) and non-raft (lane 7 to 9) fractions. Approximately 30% of the HMM form of hA3G associated with lipid rafts. Following treatment with mild nonionic detergent octyl glucoside, both the raft and non-raft fractions from HMM hA3G were subjected to the velocity gradient analysis. It shows that raft-associated hA3G was found to shift from the HMM fraction to the LMM fractions, while non-raft hA3G presented in fraction 8 at the bottom of the gradient and represented the HMM complex reported previously (Figure 2B). These data clearly demonstrate that a proportion (approximately 30%) of pelletable HMM hA3G is detergent-sensitive, which represents a LMM form of hA3G associated with lipid rafts, and the majority of pelletable hA3G appears to be mature HMM complexes.

**Figure 2:** **Steady state hA3G in the cytoplasm appears in three different forms**. **A**. 293T cells expressing HA tagged hA3G were lysed in hypotonic TE buffer. As described in Methods, P100 was prepared and treated with or without nonionic detergent octyl glucoside as indicated, then resolved by the sucrose floatation assay into the raft and non-raft proteins. Each fraction was analyzed by Western blot for the presence of hA3G, Caveolin-1 and TFR. **B**. The raft and non-raft fractions of hA3G were collected and treated with octyl glucoside, then resolved in the Opti-prep velocity gradient. Western blots of each fraction were probed with anti-HA. **C**. 293T cells expressing HA tagged hA3G were lysed in hypotonic TE buffer, and the S1 fractions were either untreated (lane 1 and 2) or treated with 0.5% Triton X-100 at 4°C (lane 3 and 4) and 37°C (lane 5 and 6), respectively. Following the ultra-centrifugation of the S1 fraction, Western blots of the P100 and S100 fractions were then probed with antibody specific for HA (top), TFR (middle), and caveolin-1 (bottom). S and P represent the S100 and P100 fractions, respectively. **D**. Fractions that respectively contain the soluble LMM (lane 1), RA LMM (lane 2) and HMM (lane 3), were subjected to immunoprecipitation with anti-HA, followed by Western blots of the immunoprecipitates probed with anti-HA, anti-RHA, and anti-Staufen, respectively.

RETRACTED

A similar result was obtained by using cellular fractionation. We treated the S1 fraction containing hA3G with 0.5% Triton X-100 (TX-100) at 37°C, which will also resulted in solubilization of lipid rafts [20,21]. Following the ultra-centrifugation of the S1 fraction, Western blots of the P100 and S100 fractions were then probed with antibody specific for HA and caveolin-1 respectively. As shown in Figure 2C, the detergent treatment resulted in total release of caveolin-1 from the P100 fraction to the S100 fraction. Simultaneously, approximately 30% of pelletable HMM hA3G (lane 6) was reduced with a corresponding increase in the soluble LMM hA3G (lane 5). In contrast, incubation of the S1 fraction with TX-100 at a low temperature (4°C), a condition that only resolves cytoplasm membrane but not lipid rafts, did not affect the distribution of either hA3G or caveolin-1. A similar result was also obtained when H9 cells were used in the same experiment as described above (data not shown).

Together these data indicate that steady state hA3G in the cytoplasm appears as three different forms: LMM hA3G (or soluble hA3G), raft-associated LMM hA3G (RA LMM hA3G) and HMM hA3G complex. Consistent with the conclusion, a co-immunoprecipitation analysis shows that Staufen and RNA helicase A (RHA), two components found in the HMM complex [14], only associated with the HMM hA3G, but not with the LMM or RA LMM hA3G (Figure 2D).

### The RA LMM hA3G acts as the precursor of the HMM hA3G complex

In an attempt to make a dynamic analysis of these three forms of hA3G, 293T cells expressing HA-tagged hA3G were labeled with [^35^S]methionine-[^35^S]cysteine for 10 min at 36 h posttransfection, followed by a chase period with cold methionine-cysteine. Aliquots of the cells were taken during the chase up to 3 hours, and then lysed hypotonically as previously described. The resultant S1 supernatant was firstly fractionated into S100 and P100 fractions. The P100 fractions were further treated with TX-100 at 37°C, and then separated by 100,000 × g centrifugation into supernatant and pellet. These fractions, which respectively contain the LMM, RA LMM, and HMM hA3G, were subjected to immunoprecipitation with anti-HA, followed by analysis of the distribution of radioactive hA3G using one-dimensional (1-D) PAGE (Figure 3A). The relative amount of radio-labeled hA3G in each fraction was determined by autoradiography and presented graphically in Figure 3B. The total amount of hA3G in each fraction was set as 100%. Results show that radio-labeled hA3G was present in the LMM and RA LMM, but not HMM fractions at 0-min of chase, i.e., after a 10-min pulse. The LMM hA3G decreased rapidly over the first 30 minutes of chase and remained stably thereafter, then reduced gradually after 2 hours post-radiolabel. In contrast, the amount of RA LMM hA3G increased during the first 30 minutes, and underwent a significant decrease thereafter. The radio-labeled hA3G in the HMM fraction increased gradually during the early time of chase, reached a peak by 1 to 2 hours and then declined. During the first 30 min chase period, the decrease of hA3G in LMM and the simultaneous increase of hA3G in RA LMM probably reflect a rapid movement of newly-synthesized hA3G to the lipid rafts. The distinct dynamics of newly-synthesized hA3G in RA LMM and HMM indicate that the RA LMM hA3G found here is not a breakdown product of the HMM hA3G complex, rather it is a distinct LMM form of hA3G. After 30 minutes chase, the amount of radio-labeled hA3G in the HMM complex increased significantly accompanied by a great reduction in newly-synthesized hA3G in RA LMM and the amount of soluble LMM hA3G remained stable. It is worthy to note that total hA3G was only reduced approximately 30% over 3 hours of chase, consistent with previous reports [22,23]. Although some LMM hA3G were degraded during the chase, the majority of LMM undergoing a significant decrease was most likely converted into the HMM form. This suggests that the RA LMM hA3G, instead of the LMM form, acts as the precursor of the HMM hA3G complex. All this reflects a dynamic course among LMM, RA LMM and HMM forms of hA3G, including a rapid movement of newly-synthesized hA3G from the LMM form to the lipid rafts, which serve as a precursor to the HMM hA3G complex.

RETRACTED

**Figure 3:** **The RA LMM hA3G acts as the precursor of the HMM complex**. 293T cells expressing hA3G were radiolabeled and chased. Aliquots of the cells were collected, and then lysed hypotonically, as described in Methods. **A**. Total cell lysate and three fractions containing LMM, RA LMM and HMM form of hA3G were subjected to immunoprecipitation with anti-HA, respectively, followed by analysis of the distribution of radioactive hA3G using one-dimensional (1-D) PAGE. **B**. The relative amount of radio-labeled hA3G in each fraction was determined by autoradiography and presented graphically. The bar graphs represent the means of results of experiments performed at least three times, and the error bars represent standard deviations.

### The correlation between the cellular distribution and viral incorporation of hA3G

Attempting to identify the cellular source of viral hA3G, we first determined if a correlation existed between the cellular distribution and viral incorporation of hA3G. We investigated the effect of a set of truncated mutations, which were described previously [6] and shown graphically in Figure 4A, upon the overall distribution of hA3G among the LMM form, the RA LMM form and the mature form of HMM hA3G complex, as described in Figure 2. The amounts of hA3G in these three forms were determined by Western blot (Figure 4B) and graphically shown in Figure 4C. It shows that hA3G missing amino acids 1-156 resulted in its failure to assemble into either the RA LMM or the mature form of the HMM complex. It is worth noting that the majority of two C-terminal deletions of hA3G resided in the RA LMM, i.e., approximately 70% of Δ157-384 formed the RA LMM and only 25% assembled into the mature HMM complex. This data suggest that the removal of the C-terminus of hA3G may impair its ability to convert the RA LMM into the mature HMM hA3G complex.

**Figure 4:** **The correlation between the cellular distribution and viral incorporation of hA3G**. **A**. Wild type and mutant hA3G. The filled rectangles represent the two zinc coordination units. The numbers represent the amino acid positions. **B**. 293T cells were co-transfected with hGag and either wild-type or mutated forms of hA3G, and the S1 fractions of the cell lysates were subjected to ultra-centrifugation and octyl glucoside treatment, resulting in the LMM, RA LMM and HMM forms of hA3G. The amounts of hA3G in the three forms were determined by Western blot. **C**. The cellular distributions of wild type and mutant hA3G are graphically shown. **D**. Western blot of cell lysates were probed with anti-HA. **E**. Western blot of virus like particle lysates probed with anti-HA. **F**. The relative amounts of mutated hA3G in the cell or viral lysates were normalized to wild-type hA3G, and then a ratio of viral to cellular hA3G was determined and used to measure its ability to be packaged into virions. The bar graphs in panel C and F represent the means of results of experiments performed at least three times, and the error bars represent standard deviations.

Next, we co-transfected 293T cells with plasmids coding for hGag and either wild-type or mutations of hA3G described above. The expression and viral incorporation of the hA3G variants were assessed by Western blots of cell and virion lysates, respectively (Figure 4D and 4E). Consistent with our previous report [6], Western blot analysis shows that hA3G missing amino acids 1-156 exhibited reduced incorporation into Gag VLPs, while the removal of the C-terminal portion of hA3G resulted in more efficient viral incorporation compared to wild type hA3G. The relative amounts of mutated hA3G in the cell or viral lysates were normalized to wild-type hA3G, and then a ratio of viral to cellular hA3G was determined and used to measure its ability to be packaged into virions (Figure 4F). A comparison of Figure 4F and Figure 4C indicates that the amount of hA3G residing in the RA LMM directly correlates with its ability to be incorporated into HIV-1. A similar quantitative change in the amounts of hA3G in the RA LMM and the virions provides further supporting evidence that the RA LMM represents the cellular source of viral hA3G.

RETRACTED

### The ability of hA3G to bind to Gag is insufficient for its incorporation into HIV-1

Several amino acid residues (i.e., W127) within the N-terminal part of the linker region play an important role in mediating the hA3G/Gag interaction. hA3G missing in this region will not likely bind to Gag, thus abolishing its incorporation into the virions [6,18,24,25]. While another mutation hA3G, Y124A, has been reported to possess the ability to bind to Gag but not to be packaged into virions [24]. To better define the role of the RA LMM in viral incorporation of hA3G, we further investigated the cellular distribution of hA3G Y124A. As shown in Figure 5A, hA3G Y124A was expressed at a similar level as wild type hA3G (left panel), whereas viral incorporation of hA3G Y124A was reduced by 3-4 folds (central panel), which is consistent with a previous report [24]. By co-immunoprecipitation analysis, similar amounts of hA3G and hA3G Y124A were detected in anti-p24 immunoprecipitates from the cell lysates (right panel), indicating that this mutant is able to interact with HIV-1 Gag as efficiently as wild-type hA3G. In contrast, viral inefficient encapsidation of W127A was mainly attributable to the loss of its interaction with HIV-1 Gag (Figure 5B). So, we further determined the distribution of wild type hA3G and hA3G Y124A among the LMM form, the RA LMM form and the mature form of HMM hA3G complex. In Figure 5C showed that the Y124A mutation, similar to the N-terminal hA3G truncations, caused a significant reduction in the RA LMM and HMM complex. This data suggest that, in addition to the ability to bind to HIV-1 Gag, the cellular distribution of hA3G is also critical for its viral incorporation.

**Figure 5:** **The ability of hA3G to bind Gag is insufficient for its incorporation into HIV-1**. 293T cells were co-transfected with plasmids coding for hGag and either hA3G Y124A (**A**) and W127A (**B**). Left panel: Western blot of cell lysates were probed with either anti-HA (top) or anti-β-actin (bottom). Middle panel: Western blot of virion lysates were probed with either anti-HA (top) or anti-p24 (bottom). Right panel: Western blots of rabbit anti-p24 immunoprecipitates were probed with either anti-HA (top) or mouse anti-p24 (bottom). **C**. Relative amounts of hA3G Y124A in the LMM, RA LMM and HMM hA3G complex were determined by Western blot and graphically presented. The bar graphs represent the means of results of experiments performed at least three times, and the error bars represent standard deviations.

RETRACTED

## Discussion

The purposes of this study are to better characterize cellular distribution of hA3G and to provide insight into the cellular source for hA3G encapsidation into HIV-1. In this work, we found that the majority of either endogenous hA3G in H9 cells, or hA3G transiently expressed in 293T cells, resided in the P100 fraction and were solely detected in the HMM fraction in a Opti-prep velocity gradient. Approximately 15% of the total hA3G appeared in the cytoplasm as a soluble form that was found in the S100 fraction after ultracentrifugation and in the LMM fraction of the velocity gradient. Using the criteria of sensitivity to the nonionic detergent octyl glucoside, we determined that the pelletable hA3G consisted of two distinct forms: RA LMM hA3G which were associated with lipid rafts and hA3G in the mature HMM complex. The HMM complex contains both Staufen and RNA helixase A, which is consistent with previous characterization of the mature HMM hA3G complex [14]. The results of a pulse-chase radiolabeling experiment revealed that the RA LMM hA3G represents the majority of newly-synthesized hA3G that associates with membrane lipid raft domains, and serves as the precursor of the HMM hA3G complex.

Although LMM hA3G can be converted to HMM complex when CD4 T cells are activated with various mitogens and cytokines [26,27], the mechanism by which hA3G is regulated to assemble into different complexes is largely unknown. Our work herein suggests two essential steps during the assembly of the HMM complex: 1) formation of the RA LMM precursor at lipid rafts and 2) conversion of this precursor into the mature HMM complex. For the first step, mutagenesis studies of hA3G revealed that the removal of amino acids 105 to 156, the linker region of hA3G, inhibited its localization at lipid raft domains to assemble the RA LMM and subsequent mature form of the HMM complex, thus resulting in a predominantly soluble LMM form of hA3G. Investigation of hA3G Y124A provides further evidence supporting the importance of the linker region for the assembly of the RA LMM and the distribution of hA3G. These data together suggest that hA3G amino acids 105-156 are required for its localization at lipid rafts where hA3G assemble into the RA LMM, the precursor of the HMM complex. A recent work has identified a novel cytoplasmic retention signal (CRS) within the linker region of hA3G [28]. The CRS residing within amino acids 113-128 is necessary and sufficient to retain hA3G in the cytoplasm. We reason that the CRS may be involved in the lipid rafts localization of hA3G and thereby restricts hA3G to the cytoplasm. Further studies are still needed to fine-map the motif within hA3G required for its cytoplasmic retention and lipid rafts localization, and to determine if a correlation exists between these two parameters.

RETRACTED

It is worthy to note that all of the hA3G C-terminal deletions tested become pelletable and no soluble LMM form was detected. One explanation for this observation is a rapid conversion of the mutants from LMM to HMM. Alternatively, other groups and we have reported that N-terminal fragments of hA3G are inherently unstable [6,29], it is thus possible that the LMM form of these mutants has been degraded rapidly and association with lipid raft may increase their stability. In addition, significant accumulation of the RA LMM form of mutants suggests that the assembly of the mature HMM hA3G complex may involve sequences further down stream of hA3G 105-156; the removal of the C-terminus of hA3G may therefore impair its ability to convert the RA LMM into the HMM complex.

Previous works have shown that reduced cellular expression of the hA3G C-terminal truncations did not result in a corresponding decrease in its viral incorporation [6]. This suggests that viruses may recruit hA3G from a particular intracellular pool, i.e., the cellular distribution of hA3G may strongly influence its viral incorporation. Indeed, the fact that hA3G Y124A is able to bind to Gag *in vitro*, but fails to be packaged into virions, suggests that some other properties of this protein, such as specific cellular localization, are also required for the interaction of these two molecules occurring *in vivo*. Khan *et al*. reported that inability of the mutant to be packaged may result from its failure to associate with lipid rafts [10]. Studies of viral incorporation of truncated hA3G show that its ability to be packaged into virions directly correlates with its concentration in the RA LMM hA3G complex (Figure 4), suggesting that the RA LMM acts as a cellular source for hA3G virion encapsidation. In agreement with this hypothesis, hA3G Y124A that is deficient in its ability to form the RA LMM and HMM complexes (the precursor and mature forms), is unable to be packaged into virions, even though it is able to interact with Gag as efficiently as wild type hA3G (Figure 5). Furthermore, the movement of newly-synthesized hA3G to lipid raft domains to rapidly form the RA LMM is consistent with a previous finding that hA3G is incorporated into the virion shortly after its synthesis in cytoplasm [17]. These data together indicate that the RA LMM hA3G complex acts as the cellular source for its virion encapsidation.

RETRACTED

Since HIV-1 Gag concentrates in the multivesicular bodies (MVB)/late endosomal compartments enriched in lipid rafts during virion assembly, one explanation for the role of the RA LMM hA3G in the incorporation is the localization in lipid rafts, where both Gag and hA3G concentrate, thereby interacting with each other. In agreement with the hypothesis, hA3G has been shown to associate with intracellular membrane rafts, and more specifically, late endosomal vesicles [5].

## Conclusions

This work thus provides the first evidence for the existence of RA LMM hA3G complex and leads toward a better understanding of the regulation of hA3G regarding its antiviral and cellular functions. The potential implications of this work for the development of anti-HIV therapeutics include either enhanced viral incorporation of hA3G by accumulation of the RA LMM complex, or increased accumulation of the LMM complex by blocking its localization at lipid rafts, which may produce a Vif-resistant post-entry inhibition on HIV-1 replication found in resting T cells.

## Methods

### Plasmid construction

The hGag plasmid, which encodes the HIV-1 Gag sequence, produces mRNA whose codons have been optimized for mammalian codon usage, and was a kind gift from G Nabel, NIH [30]. The construction of wild-type and mutant forms of hA3G has been previously described [6]. hA3G Y124A was constructed using a site-directed mutagenesis kit (Stratagene) and confirmed by sequencing.

### Cell, transfection and virus purification

The culture and transfection of HEK-293T cells with these plasmids using Lipofectamine 2000 (Invitrogen, Carlsbad, California), and the isolation of virions 48 h posttransfection from the cell supernatant, were done as previously described [6,31]. Unless stated otherwise, 293T cells were transfected with 1 μg of hGag and 1 μg of plasmid coding for wild type or mutant forms of hA3G. The total amount of plasmid DNA used for transfection was kept constant in controls by replacing plasmid coding for hA3G with the empty vector, pcDNA3.1.

### Protein Analysis

Cellular and viral proteins were extracted with RIPA buffer (10 mM Tris, pH 7.4, 100 mM NaCl, 1% sodium deoxycholate, 0.1% SDS, 1% NP40, 2 mg/ml aprotinin, 2 mg/ml leupeptin, 1 mg/ml pepstatin A, 100 mg/ml PMSF). Equal amounts of protein (determined by a Bio-Rad assay) were analyzed by SDS PAGE (10% acrylamide), followed by blotting onto nitrocellulose membranes (Amersham Pharmacia). Western blots were probed with the following antibodies that are specifically reactive with: HIV-1 capsid (Zepto Metrocs Inc.), HA, TFR (Invitrogen) and caveolin-1 (Santa Cruz Biotechnology Inc.), β-actin (Sigma), RNA helicase (a gift from Chen Liang [32]), Staufen (a gift from Andrew Mouland [33]). Detection of proteins was performed by enhanced chemiluminescence (NEN Life Sciences Products), using as secondary antibodies anti-mouse and anti-rabbit, both obtained from Amersham Life Sciences. Bands in Western blots were quantitated using the ImageJ 1.35 s automated digitizing system (NIH).

RETRACTED

### Subcellular fractionation

293T cells were lysed 48 h post-transfection at 4°C in hypotonic medium; lysis was done by Dounce homogenization in 1.0 ml of hypotonic TE buffer (20 mM Tris-HCl, pH 7.4, 1 mM EDTA, 0.01% ß-mercaptoethanol) supplemented with protease inhibitor cocktail (Complete; Boehringer Mannheim) and RNase inhibitors (Ambion). The cell homogenate was then centrifuged at 1,500 × *g *for 30 minutes to remove nuclei and unbroken cells. The supernatant (S1) was then centrifuged for 1 h at 100,000 × *g *in an SW55Ti rotor (Beckman, Columbia, Md.) at 4°C, resulting in the supernatant (S100) and the pellet (P100). To resolve cytoplasmic membrane or lipid rafts, the S100 and the P100 suspended in 1 ml of hypotonic TE buffer was incubated with 0.5% Triton X-100 at 4°C or 37°C for 15 minutes, respectively.

Resolution of hA3G into the LMM and HMM forms was performed, using a 4-35% discontinuous Opti-prep velocity gradient. This gradient was prepared in advance by layering 0.5 ml of 35%, 0.5 ml of 30%, 0.5 ml of 25%, 1.5 ml of 20%, 0.5 ml of 15%, 0.5 ml of 10%, and 0.5ml of 4% Opti-prep from bottom to top. 0.5 ml of the S1, S100 or the P100 re-suspended in hypotonic TE buffer was layered on top of the gradient, and then centrifuged at 100,000 × *g *in a Beckman SW55Ti rotor for 1 h at 4°C. Nine fractions (0.5 ml) were collected and diluted with an equal volume of 2× TNT, and each fraction was subjected to Western blot or immunoprecipitation analysis.

### Memberane floatation assay (raft association)

293T cells expressing HA tagged hA3G were lysed and fractionated into S100 and P100 as described above. The pellet P100 was resuspended in TNE buffer (100 mM Tris-HCl, 600 mM NaCl, 16 mM EDTA, supplemented with protease inhibitor cocktail and RNase inhibitors) containing either 0.5% Triton X-100 or 0.5% nonionic detergent *n*-octyl-*β*-D-glucopyranoside (octyl glucoside). Following mixed with 85.5% sucrose (w/v) in TNE lysis buffer to obtain 73% sucrose (w/v), samples were placed at the bottom of ultracentrifuge tubes, and overlaid with 65% (w/v) sucrose and 10% sucrose (w/v) in TNE lysis buffer. Then samples were centrifuged at 4°C in a SW55 rotor for 16 hours at 35,000 rpm to obtain raft and non-raft associated fractions [18,34]. Nine equal fractions were collected from the top, followed by analysis of Western blot.

RETRACTED

### Immunoprecipitation assay

293T cells from 100 mm plates were collected 48 hours post transfection, and lysed in 500 μl TNT buffer (20 mM Tris-HCl pH 7.5, 200 mM NaCl, 1% Triton X-100). Insoluble material was pelleted at 1800 × g for 30 minutes. Equal amounts of protein were incubated with 5 μl HA (or p24)-specific antibody for 16 hours at 4°C, followed by the incubation with protein A-Sepharose (Pharmacia) for two hours. The immunoprecipitate was then washed three times with TNT buffer and twice with phosphate-buffered saline (PBS). After the final supernatant was removed, 30 μl of 2X sample buffer (120 mM Tris HCl, pH 6.8, 20% glycerol, 4% SDS, 2% β-mercaptoethanol, and 0.02% bromphenol blue) was added, and the precipitate was then boiled for 5 minutes. After microcentrifugation, the resulting supernatant was analyzed using Western blots, as previously described [35].

### Pulse-chase radiolabeling experiments

Transfected 293T cells were labeled 36 h posttransfection with 400 μCi of [^35^S]methionine-[^35^S]cysteine for 15 minutes and then chased for various lengths of time in Dulbecco modified Eagle medium containing 10% fetal bovine serum and 100 μM cysteine and methionine. After being washed, the cells were lysed hypotonically by Dounce homogenization in 1 ml of hypotonic TE buffer at 4°C, and the cell lysates were centrifuged at 1,500 × *g *for 30 min to remove nuclei and unbroken cells. The resulting S1 supernatant (1 ml) was fractionated into S100 and P100 fractions by centrifuging for 1 h at 100,000 × *g *in SW55Ti rotor at 4°C. The P100 fractions were further treated with octyl glucoside, and then separated by 100,000 × g centrifugation into a supernatant and pellet which contain RA LMM and HMM hA3G, respectively. The immunoprecipitation with anti-HA was performed, followed by analysis of the distribution of radioactive hA3G using one-dimensional (1-D) PAGE and autoradiography.

## Competing interests

The authors declare that they have no competing interests.

## Authors' contributions

First three authors contributed equally to this work. JM, XYL and JX have made equal contributions to conception and design, acquisition of data, and analysis and interpretation of data. JM was involved in drafting the manuscript. QZ, ZLL and PPJ carried out the mutation construction. FG, LYY and XFY participated in the design of the study and performed the statistical analysis. LXZ and JDJ were involved in revising the manuscript and helping to draft the manuscript. SC supervised the project and commented on the manuscript. All authors read and approved the final manuscript.
